The article "Application Effect Analysis of Clinical Nursing Pathway in the Care of Neonatal Hypoxic-Ischemic Encephalopathy" was retracted in 2023. Reasons: unreliable results or conclusions; concerns about the data; concerns about the peer review; concerns about the citations.

# Application Effect Analysis of Clinical Nursing Pathway in the Care of Neonatal Hypoxic-Ischemic Encephalopathy

**DOI:** 10.1155/2022/9379361

**Published:** 2022-06-16

**Authors:** Xiaoyu Zhang, Hai Wang

**Affiliations:** Department of Obstetrics, The First Affiliated Hospital of Heilongjiang University of Chinese Medicine, Harbin, 150040 Heilongjiang, China

## Abstract

This research focuses on the effectiveness of the clinical nursing pathway (CNP) in the treatment of infant hypoxic-ischemic encephalopathy (NHIE). This research enrolled 120 cases of NHIE admitted to the First Affiliated Hospital of Heilongjiang University of Chinese Medicine, including 70 cases (research group, the Res) who received CNP intervention and 50 cases (control group, the Con) treated by routine nursing pathway intervention. The psychomotor development index (PDI), mental development index (MDI), neurodevelopment (ND), physique growth, and incidence of adverse events (AEs) were recorded and analyzed. The results identified that in comparison with the Con (1) the PDI and MDI were obviously better in the Res 6 months postintervention; (2) the Res had significantly superior ND of behavioral capacity, passive tone, active tone, primitive reflex, and general assessment 1 month after intervention, as well as physical development of body weight, height, and head circumference after 40 days of birth, (3) the incidence of total AEs within 40 days was statistically lower in the Res. As a result, CNP is considerably superior to the traditional nursing pathway in the treatment of NHIE, and it merits clinical promotion.

## 1. Introduction

Birth asphyxia is the most common risk factor for early neonatal death, followed by premature delivery, low birth weight, and infection [1]. The exploration of the pathological mechanism of neonatal asphyxia found that hypoxia and ischemia can make the nutrition and energy supply of the neonatal brain abnormal, which in turn leads to neuronal cell death, cell dysfunction, and neurodevelopmental defects [2]. Neonatal hypoxic-ischemic encephalopathy (NHIE) is one of the serious complications of perinatal asphyxia, and its etiology is related to impair ND [3]. According to statistics, about a quarter of NHIE cases will die during the neonatal period, and another quarter may develop long-term sequelae such as cerebral palsy, epilepsy, and sensory disturbance, which seriously compromise the healthy growth of children's body and mind [4]. Choosing appropriate and effective treatment methods is crucial to improve the prognosis of NHIE children, and the postnatal care of neonates with hypoxic-ischemic encephalopathy (HIE) is also critical [5, 6]. Accordingly, we herein discuss the application effect of nursing intervention for NHIE, aiming at providing clinical reference for improving the neurological and physical development of HIE children, which is of positive significance for improving the prognosis of such neonates.

As far as the healthy development of families and even the country is concerned, improving the survival rate and long-term neurodevelopmental outcome of children with HIE has huge implications [7]. At present, routine nursing mainly focuses on targeted treatment or nutritional support, which has no significant effect on improving neither the ND nor the long-term ND outcome of HIE children [8]. The clinical nursing pathway (CNP) is mainly aimed at helping children with HIE improve their ND by providing the children's family members with disease introduction, oxygen guidance, and rehabilitation direction and giving sensory stimulation training to children during their hospitalization [9]. CNP is currently widely utilized in a variety of conditions, including advanced schistosomiasis ascites, acute bronchial asthma, and acute cerebral hemorrhage, with the benefits of lower mortality, less adverse reactions, and faster resolution of clinical symptoms and indications [10–12]. In addition, CNP has been proved to facilitate neurological recovery and improve the curative effect and prognosis of childhood diseases (e.g., nephropathy) [13, 14]. We believe that CNP is effective and has positive significance for the ND and physique growth of HIE children. We hereby compare the application effect of CNP with routine nursing in the care of NHIE and report it.

This study is unique in that it examines the effectiveness and dependability of CNP in the care of NHIE from a variety of viewpoints, including PDI, MDI, ND, physical growth, and safety, providing fresh insights into nursing techniques for NHIE. There are various limitations to this study that will need to be addressed in future research.

## 2. Data and Methods

### 2.1. General Data

This research enrolled 120 cases of NHIE treated in the First Affiliated Hospital of Heilongjiang University of Chinese Medicine between December 2017 and December 2020 and assigned them into a research group (the Res, *n* = 70) receiving CNP intervention and a control group (the Con, *n* = 50) treated by routine nursing pathway intervention. The male-to-female ratio and the mean gestational age in the Res were 32 : 38 and 39.17 ± 2.89 years, respectively, while in the Con they were 22 : 28 and 39.43 ± 2.73 years, respectively. Inclusion criteria: diagnosis of HIE; no placenta residue during delivery; neonatal birth weight: 3-5 kg; voluntary participation of the neonate's family members, with the consent form provided; no maternal genetic diseases that can pass on to the baby. Exclusion criteria: severe multiple organ dysfunction, hematopathy or infectious diseases, neurologic disorders, other congenital diseases, and incomplete clinical data. This research was ethically ratified by the First Affiliated Hospital of Heilongjiang University of Chinese Medicine.

### 2.2. Nursing Methods

A standard nursing pathway intervention was given to the Con. Nurses treated hypoglycemia, hypotension, and acidosis; administered oxygen; and cleansed the respiratory secretions of infants on a regular basis to maintain the respiratory tract clear. Anti-infection treatment or nutritional support was given according to the presence of infection and malnutrition. Nursing staff also attached special importance to the mental state, vital signs, and skin color of neonates.

#### 2.2.1. CNP Was Implemented in the Res in addition to Routine Nursing

(1) On the first day of admission, the neonates' families were introduced to the environmental function of the ward, the relevant matters that doctors and nurses were responsible for, and the work schedule and safety system. Besides, health education, etiology, and clinical symptoms of HIE as well as matters needing attention during hospitalization were disseminated to the neonates' families. (2) On the second day of admission, related knowledge of oxygen use was introduced to the neonates' families, and guidance was given to them so that they could understand the knowledge of oxygen inhalation and the appropriate way of oxygen supply. Family members were also told to remove respiratory secretions as soon as possible to keep the respiratory tract clear and avoid suffocation while sleeping. (3) On day 3 after admission, some children with high fever were treated with mild hypothermia, and health education and publicity were given to the families of such children so that the families could have a certain understanding of the precautions when the children were cooled down and maintained. (4) On the fourth day of admission, children's sensory stimulation was strengthened for passive gymnastics training. (5) On day 5 after admission, family members were instructed in rehabilitation training, as early motor and perception training is helpful to promote the recovery of brain function. By patiently answering the illness of the newborns to the families, the nursing staff gained the trust and understanding of family members. In addition, parents were instructed to master the rehabilitation training measures during the convalescence period, so as to obtain parental cooperation and enhance their compliance with the regular follow-up.

### 2.3. Endpoints

#### 2.3.1. Mental Development Index (PDI) and Mental Development Index (MDI) [15]

The scores of these two indicators are above 120 points for excellent, 110-119 points for upper-middle intelligence, 90-109 points for moderate intelligence, 80-89 points for middle-lower points, 70-79 points for critical state, and below 69 points for mental retardation.

#### 2.3.2. ND

The neonates were scored for their neurodevelopmental status using the Neonatal Behavioral Neurological Assessment (NBNA) [16] from the aspects of behavior, passive tone, active tone, primitive reflex, and general assessment. The score was proportional to the ND of children.

#### 2.3.3. Physique Growth

It was evaluated by measuring the weight gain, height gain, and head circumference growth of children.

#### 2.3.4. Incidence of Adverse Events (AEs)

The cases of anemia, emaciation, malnutrition, growth retardation, cough and vomiting, hypotension, intracranial hypertension, and other AEs were observed and recorded.

### 2.4. Statistical Processing

The software used for data analysis and image description was SPSS *v*23.0 and GraphPad Prism *v*8.0, respectively. For counting data described in the form of number of cases/percentages (*n*(%)), either the chi-square test or the chi-square test with continuity correction (applied when the theoretical frequency in the chi-square test was less than 5) was used for intragroup comparisons. Mean ± standard deviation (SD) was used to represent the measurement data, and the statistical methods for intergroup and intragroup (before and after treatment) comparisons were independent samples *t*-test and paired *t*-test, respectively. *P* < 0.05 is regarded as the difference with statistical significance.

## 3. Results

### 3.1. General Data

The two cohorts of patients were comparable in age, gestational age, head circumference, weight, natural delivery, and symptoms (*P* > 0.05) (Table 1).

### 3.2. Comparative Analysis of PDI and MDI between Two Groups of Patients

We evaluated the psychomotor development (PMD) and intelligence development of the two groups of patients by PDI and MDI, respectively. The data showed no evident difference in PDI and MDI between groups before nursing (*P* > 0.05) and notably elevated parameters after nursing, especially in the Res, with statistical significance (*P* < 0.05) (Figure 1).

### 3.3. ND of Two Groups of Patients

We analyzed neonates' ND with the NBNA scale. The data identified significantly enhanced behavioral capacity, passive tone, active tone, primitive reflex, and general assessment in both groups after nursing; moreover, in comparison with the Con, the five indexes were higher in the Res at 2 weeks and 1 month of birth, with statistical significance (*P* < 0.05) (Figure 2).

### 3.4. Physique Growth of Two Groups of Patients

We evaluate the physique growth of newborns through three indicators: weight gain, height gain, and head circumference growth. The Res had much higher weight gain, height rise, and head circumference growth than the Con, with statistical significance (*P* < 0.05) (Figure 3).

### 3.5. Incidence of AEs in Two Groups

We observed and compared the incidence of AEs to evaluate the influence of different nursing intervention methods on AEs. The results identified a markedly lower incidence of AEs in the Res versus the Con (8.58% *vs.* 32.00%, *P* < 0.05) (Table 2).

## 4. Discussion

HIE is a brain dysfunction related to oxygenation and blood flow insufficiency [17]. Our research has confirmed that CNP has a good application effect in the care of NHIE, which can significantly promote the PMD, intelligence development, ND, and physique growth of HIE children with a favorable safety profile.

Traditional nursing intervention has been shown to have several limitations, as the nursing procedure's basic thought cannot fully adjust to illness development or address patients' main clinical demands [18]. CNP, on the other hand, is a modern nursing model that emphasizes postadmission cognition, treatment, and rehabilitation guidance for hospitalized patients; it requires nurses to have professional knowledge reserves, and it meets the needs of patients by formulating reasonable and predictable nursing programmes [19]. In our study, the children who received routine nursing pathway were set as the Con, and those who received CNP were taken as the Res. The research data showed significantly elevated PDI and MDI scores in the Res after nursing, which was statistically higher than the Con, indicating that the CNP can significantly improve the PMD and intellectual development of patients. In terms of ND, the behavioral capacity, passive tone, active tone, primitive reflex, and general assessment in the Res were statistically better than those before treatment and the Con after nursing, suggesting that the CNP has significant positive significance for the ND of HIE children. Physically, more evident weight gain, height gain, and head circumference growth were observed in the Res, demonstrating that CNP is helpful to promote the physique growth of children with HIE. CNP's intervention in children's movement and perception training, as well as the guidance of rehabilitation training for children's family members, is credited with increasing children's nerve, intelligence, and motor development [20]. Finally, we assessed the safety of neonates in both groups and discovered that they were mostly malnourished, growth retarded, and emaciated. In addition, the Res had a significantly decreased overall incidence of AEs, implying that the CNP provides some assurance of postpartum child safety.

## 5. Conclusion

The novelty of this study lies in the analysis of the effectiveness and reliability of CNP in the care of NHIE from multiple perspectives of PDI, MDI, ND, physique growth, safety, etc., which provides new insights for the choice of nursing strategies for NHIE. This study also has several limitations, which need to be gradually addressed in future research. First, given the limited cases included, it is necessary to increase the sample size to improve the accuracy and universality of the research results. Second, there is no long-term follow-up. Supplementary examination of this feature can be used to assess children's long-term neurodevelopmental outcomes, which can help to enhance their long-term prognosis. Third, if the analysis of risk factors affecting neurological development of HIE children can be increased; the nursing strategy can be further optimized.

Evidence from this study shows that while reducing the incidence of AEs, CNP is beneficial to improve the PMD, intellectual development, ND, and physique growth of children with HIE, which provides new cognition for the management of NHIE and helps to improve the prognosis of children.

## Figures and Tables

**Figure 1:** PDI and MDI of two groups of patients. (a) Comparative analysis of PDI between two groups of patients. (b) Comparative analysis of MDI between two groups of patients. Note: ^∗∗^*P* < 0.01.

**Figure 2:** Neurodevelopment of two groups of patients. (a) Behavioral capacity of two groups of patients at 2 weeks and 1 month of birth. (b) Passive muscle tone of two groups of patients at 2 weeks of birth and 1 month of birth. (c) Active muscle tone of two groups of patients at 2 weeks and 1 month of birth. (d) The primitive reflex of two groups of patients at 2 weeks and 1 month of birth. (e) The general reflex of two groups of patients at 2 weeks and 1 month of birth. Note: ^∗^*P* < 0.05; ^∗∗^*P* < 0.01.

**Figure 3:** Physique growth of patients in two groups. (a) Weight gain of neonates in the two groups after 40 days of birth. (b) Height gain of neonates in the two groups after 40 days of birth. (c) Head circumference growth of neonates in the two groups after 40 days of birth. Note: ^∗∗^*P* < 0.01.

**Table 1:** Baseline data of patients in the two groups (*n*(%), mean ± SD).

Variables	*n*	Control group (*n* = 50)	Research group (*n* = 70)	*χ* ^2^/*t*	*P*
Gender				0.035	0.85
Male	54	22 (44.00)	32 (45.71)		
Female	66	28 (56.00)	38 (54.29)		
Gestational age (weeks)	120	39.43 ± 2.73	39.17 ± 2.89	0.504	0.62
Head circumference (cm)	120	33.90 ± 3.16	33.54 ± 3.21	0.610	0.54
Weight (kg)	120	3.41 ± 0.45	3.36 ± 0.42	0.624	0.53
Natural delivery				0.403	0.52
Yes	37	17 (34.00)	20 (28.57)		
No	83	33 (66.00)	50 (71.43)		
Symptoms				0.040	0.98
Seizures or hyperexcitability	35	15 (30.00)	20 (28.57)		
Lethargy	54	22 (44.00)	32 (45.71)		
Indifference or coma	31	13 (26.00)	18 (25.72)		

**Table 2:** Incidence of adverse events in two groups of patients (*n*(%)).

Categories	Control group (*n* = 50)	Research group (*n* = 70)	*χ* ^2^ value	*P* value
Anemia	2 (4.00)	1 (1.43)	—	—
Emaciation	3 (6.00)	1 (1.43)	—	—
Malnutrition	4 (8.00)	1 (1.43)	—	—
Growth retardation	3 (6.00)	2 (2.86)	—	—
Cough and vomiting	1 (2.00)	0 (0.00)	—	—
Hypotension	2 (4.00)	0 (0.00)	—	—
Intracranial hypertension	1 (2.00)	1 (1.43)	—	—
Total	16 (32.00)	6 (8.58)	10.693	0.001

## Data Availability

The simulation experiment data used to support the findings of this study are available from the corresponding author upon request.

## References

[1] Olack B., Santos N., Inziani M. (2021). Causes of preterm and low birth weight neonatal mortality in a rural community in Kenya: evidence from verbal and social autopsy. *BMC Pregnancy Childbirth*.

[2] Koehn M., Chen X., Logsdon F., Lim P., Stonestreet S. (2020). Novel neuroprotective agents to treat neonatal hypoxic-ischemic encephalopathy: inter-alpha inhibitor proteins. *International Journal of Molecular Sciences*.

[3] Bersani I., Piersigilli F., Gazzolo D. (2021). Heart rate variability as possible marker of brain damage in neonates with hypoxic ischemic encephalopathy: a systematic review. *European Journal of Pediatrics*.

[4] Dumbuya S., Chen L., Wu Y., Wang B. (2021). The role of G-CSF neuroprotective effects in neonatal hypoxic-ischemic encephalopathy (HIE): current status. *Journal of Neuroinflammation*.

[5] Kane A., Vezina G., Chang T. (2021). Early versus late brain magnetic resonance imaging after neonatal hypoxic ischemic encephalopathy treated with therapeutic hypothermia. *J Pediatr.*.

[6] Cooper J. (2011). Induced hypothermia for neonatal hypoxic-ischemic encephalopathy: pathophysiology, current treatment, and nursing considerations. *Neonatal Network*.

[7] Wang Z., Zhang P., Zhou W. (2021). Neonatal hypoxic-ischemic encephalopathy diagnosis and treatment: a national survey in China. *BMC Pediatrics*.

[8] Synnes R., Petrie J., Grunau E. (2022). Canadian Neonatal Follow-Up Network Investigators. Family integrated care: very preterm neurodevelopmental outcomes at 18 months. *Archives of Disease in Childhood - Fetal and Neonatal Edition*.

[9] Li W., Gao J., Wei S., Wang D. (2016). Application values of clinical nursing pathway in patients with acute cerebral hemorrhage. *Experimental and Therapeutic Medicine*.

[10] Mei-Zhi Y., Jing-Ru S., Tao C., Xiao-Yu Z., Liang-Cai H., Jia-Song W. (2016). Application of clinical nursing path integrated with holistic nursing in advanced schistosomiasis patients with ascites. *Zhongguo Xue Xi Chong Bing Fang Zhi Za Zhi*.

[11] Fu S., Han H., Fan C., Jiang Y. (2020). Clinical nursing pathway improves the nursing satisfaction in patients with acute cerebral hemorrhage: a randomized controlled trial protocol. *Medicine*.

[12] Gao F., Wang H., Wang H. (2021). Study on the effect of one-stop service combined with clinical nursing path on patients with acute bronchial asthma. *American Journal of Translational Research*.

[13] Yang Y., Mu A., Wang Y. (2021). Early path nursing improves neurological function recovery in patients with intracerebral hemorrhage: protocol for a randomized controlled trial. *Medicine*.

[14] Yu X., Han Y. (2021). Effect assessment of evidence-based nursing in combination with clinical nursing pathway on nephrotic syndrome care in children: a protocol for systematic review and meta-analysis. *Medicine*.

[15] Nichols R., Rundle G., Factor-Litvak P. (2020). Prepregnancy obesity is associated with lower psychomotor development scores in boys at age 3 in a low-income, minority birth cohort. *Journal of Developmental Origins of Health and Disease*.

[16] Liu C., Messerlian C., Chen J. (2021). Trimester-specific associations of maternal exposure to disinfection by-products, oxidative stress, and neonatal neurobehavioral development. *Environment International*.

[17] Wilson A., Fell B., Hawken S. (2019). Association between newborn screening analytes and hypoxic ischemic encephalopathy. *Scientific Reports*.

[18] Adlbrecht L., Nemeth T., Frommlet F., Bartholomeyczik S., Mayer H. (2021). Engagement in purposeful activities and social interactions amongst persons with dementia in special care units compared to traditional nursing homes: an observational study. *Scandinavian Journal of Caring Sciences*.

[19] Liu X., Wang L., Zhang K. (2021). Study on clinical nursing pathway to promote the effective implementation of sepsis bundle in septic shock. *European Journal of Medical Research*.

[20] Zhang Y., Zhang L., Li Y. (2016). Computed tomography diagnosis of neonatal hypoxic ischemic encephalopathy combined with intracranial hemorrhage and clinical nursing treatment. *Journal of Biological Regulators and Homeostatic Agents*.

